The article "Alpha-synuclein contributes to malignant progression of human meningioma via the Akt/mTOR pathway" was published in 2016. Journal: Cancer Cell Int.

# Alpha-synuclein contributes to malignant progression of human meningioma via the Akt/mTOR pathway

**DOI:** 10.1186/s12935-016-0361-y

**Published:** 2016-11-15

**Authors:** Yiqin Ge, Kan Xu

**Affiliations:** Department of Neurosurgery, Putuo Hospital, Shanghai University of Traditional Chinese Medicine, No.164 Lanxi Road, Shanghai, 200062 China

**Keywords:** Akt/mTOR signaling, α-Synuclein, Growth, Invasion, Meningioma

## Abstract

**Background:**

The aim of this study is to explore the expression of alpha-synuclein (α-synuclein) in benign, atypical, and anaplastic meningiomas and determine its role in the malignant progression of meningiomas.

**Methods:**

Expression of α-synuclein was measured in 44 meningioma samples by real-time PCR analysis. The effects of overexpression or knockdown of α-synuclein on meningioma cell growth, invasiveness, and tumorigenicity were determined.

**Results:**

Atypical and anaplastic meningiomas displayed significantly greater levels of α-synuclein mRNA, relative to benign tumors. Depletion of α-synuclein decreased cell proliferation and colony formation and promoted apoptosis in IOMM-Lee meningioma cells, whereas overexpression of α-synuclein facilitated cell proliferation and colony formation in CH-157MN meningioma cells. Silencing of α-synuclein attenuated IOMM-Lee cell migration and invasion. In contrast, ectopic expression of α-synuclein increased the invasiveness of CH-157MN cells. In vivo studies further demonstrated that downregulation of α-synuclein significantly retarded meningioma growth in nude mice. At the molecular level, the phosphorylation levels of Akt, mTOR, p70S6K and 4EBP were significantly decreased in α-synuclein-depleted IOMM-Lee cells.

**Conclusions:**

In conclusion, α-synuclein upregulation contributes to aggressive phenotypes of meningiomas via the Akt/mTOR pathway and thus represents a potential therapeutic target for malignant meningiomas.

## Background

Meningiomas are mesenchymal tumors that account for ~30% of all primary intracranial tumors [1]. Most meningiomas are benign tumors of World Health Organization (WHO) grade I. However, up to 20% of meningiomas have aggressive behaviors, which are classified as atypical WHO grade II or anaplastic WHO grade III [2]. The Akt/mTOR pathway has been suggested to be involved in the pathogenesis of meningiomas [3, 4]. However, the molecular mechanisms underlying the malignant progression of meningiomas are still elusive.

Alpha-synuclein (α-synuclein) is a soluble presynaptic protein belonging to the synuclein protein family. It is well known that α-synuclein can form insoluble fibril aggregates and play a pathogenic role in Parkinson’s disease (PD) [5]. In addition to expression in nervous tissues, α-synuclein is expressed in other tissue types such as melanomas [6–8]. It was found that α-synuclein is abundantly presented in primary and metastatic melanomas, but undetectable in non-melanocytic cutaneous carcinoma and normal skin [6]. There is evidence that α-synuclein differentially regulates the synthesis of melanin in melanoma and dopaminergic neuronal cells, consequently affecting cell susceptibility to ultra-violet radiation-induced injury [8]. A previous study has demonstrated that α-synuclein is expressed in a variety of brain tumors, but not in benign meningiomas [9]. However, the expression and biological relevance of α-synuclein in the malignant progression of meningiomas are not clarified.

The article "Alpha-synuclein contributes to malignant progression of human meningioma via the Akt/mTOR pathway" was published in 2016. Journal: Cancer Cell Int.

In this study, we compared the expression of α-synuclein in atypical and anaplastic meningiomas versus benign tumors and explored the roles of α-synuclein in regulating the aggressive phenotypes of meningiomas.

## Methods

### Tissue samples

A total of 44 meningioma specimens (18 benign, 17 atypical, and 9 anaplastic meningiomas) were obtained from patients who underwent surgery at Department of Neurosurgery of Shanghai University of Traditional Chinese Medicine (Shanghai, China). Tumor tissues were immediately frozen in liquid nitrogen and stored at −80 °C until analysis. All cases were pathologically diagnosed. Tumors were classified according to the 2007 WHO classification system [10].

### Cell culture

Primary human meningeal cells were purchased from ScienCell (Carlsbad, CA, USA). IOMM-Lee and CH-157MN meningioma cell lines were obtained from the Shanghai Institute of Cell Research (Shanghai, China). Cells were cultured in high-glucose Dulbecco’s modified Eagle medium (DMEM) with 10% fetal bovine serum (FBS), 100 μg/mL streptomycin, and 100 U/mL penicillin (Invitrogen, Carlsbad, CA, USA).

### Quantitative real-time PCR (qRT-PCR) analysis

Total RNA from tumor tissues and cells was extracted using TRIzol reagent (Takara, Dalian, China) following the manufacturer’s protocol. Reverse transcription was completed with random primers using the Superscript III Reverse Transcriptase Kit (Invitrogen, Carlsbad, CA, USA). Real-time PCR was performed on an ABI7900 Real-Time PCR System (Applied Biosystems, Foster City, CA, USA) using SYBR Green RT-PCR kit (QIAGEN, Valencia, CA, USA). The PCR primers are as follows [11]: α-synuclein: forward, 5′-GCCAAGGAGGGAGTTGTGGCTGC-3′ and reverse, 5′-CTGTTGCCACACCATGCACCACTCC-3′; β-actin: forward, 5′-TCTACAATGAGCTGCGTGTG-3′ and reverse, 5′-GGTGAGGATCTTCATGAGGT-3′. The relative α-synuclein mRNA level was determined after normalization against that of β-actin.

The article "Alpha-synuclein contributes to malignant progression of human meningioma via the Akt/mTOR pathway" was published in 2016. Journal: Cancer Cell Int.

### Plasmids and transfections

Small hairpin RNA (shRNA) targeting human α-synuclein gene and negative control shRNA were purchased from Santa Cruz Biotechnology (Santa Cruz, CA, USA). For generation of α-synuclein-expressing plasmid, full-length human α-synuclein cDNA was amplified by PCR and cloned into pcDNA3.1(+) vector (Invitrogen). Cell transfections were performed using HiPerfect Transfection reagent (Qiagen, Hilden, Germany). After incubation for 24 h, cells were subjected to further analyses. For generation of stable clones, IOMM-Lee cells transfected with α-synuclein shRNA or control shRNA were selected with puromycin (2 μg/mL; Sigma-Aldrich) for 3 days.

### BrdU incorporation assay

Cell proliferation was assessed by 5-bromo-2′-deoxyuridine (BrdU) incorporation assay using the Cell Proliferation ELISA, BrdU (colorimetric) kit (Roche Applied Science, Indianapolis, IN, USA). In brief, cells were labeled using 10 μM BrdU and incubated overnight at 37 °C. The cells were then fixed and re-incubated with anti-BrdU antibody for 2 h at room temperature. The substrate solution was added and the reaction product was quantified by measuring the absorbance at 450 nm.

### Apoptosis analysis

For analysis of apoptosis, cells were fixed in 70% ethanol and incubated with propidium iodide and Annexin-V for 30 min. Stained cells were analyzed on a flow cytometer (Becton–Dickinson Biosciences, San Jose, CA, USA).

### Colony formation assay

Transfected cells were seeded onto six-well plates at a low density (600 cell per well) and cultured for 10 days. Colonies were fixed, stained with 0.1% crystal violet (Sigma-Aldrich), and counted.

### In vitro wound-healing assay

Cell migration capacity was evaluated using in vitro wound-healing assay, as described previously [12]. In brief, cells were seeded onto six-well plates and allowed to grow to confluence. The cell monolayer was scratched with a 100-μL pipette tip. After washing, the cell culture was incubated for 24 h. The percentage of wound closure was determined under a microscope. This assay was repeated three times.

### Transwell invasion assay

Cells in serum-free medium (1 × 10^5^ cells/well) were plated onto the upper chamber pre-coated with Matrigel (Becton–Dickinson Biosciences). The lower chamber was added with DMEM containing 10% FBS. After incubation for 24 h, cells that had invaded through the Matrigel were stained with 0.1% crystal violet and counted.

### Animal experiments

Eight 6–8-week-old nude mice (Shanghai Laboratory Animal Center, Chinese Academy of Sciences, Shanghai, China) were used for tumorigenic studies. IOMM-Lee cells stably transfected with α-synuclein shRNA or control shRNA were subcutaneously injected into nude mice (n = 4; 4 × 10^6^ cells/mouse). Tumor volume was determined every 5 days. At 25 days after cell injection, mice were sacrificed and xenograft tumors were removed and weighed.

The article "Alpha-synuclein contributes to malignant progression of human meningioma via the Akt/mTOR pathway" was published in 2016. Journal: Cancer Cell Int.

### Western blot analysis

Protein extracts from tumor tissues and cells were prepared in radioimmunoprecipitation assay (RIPA) buffer containing protease inhibitors (Sigma-Aldrich). Protein samples were separated by sodium dodecyl sulphate–polyacrylamide gel electrophoresis and transferred onto nitrocellulose membranes. Primary antibodies (1:500 dilution) used here are as follows: anti-Akt, anti-Akt (ser473), anti-mTOR, anti-phospho-mTOR (Ser2448), anti-phospho-p70S6K1 (Thr389), anti-p70S6K1, anti-phospho-4EBP (Thr37/46), anti-4EBP (Cell Signaling Technology, Beverly, MA, USA), anti-α-synuclein (Abcam, Cambridge, MA, USA), and anti-β-actin (Sigma-Aldrich). Blots were developed with an enhanced chemiluminescence system (GE Healthcare Biosciences, Piscataway, NJ, USA). Densitometric analysis of the blots were performed using the Quantity One software (Bio-Rad Laboratories, Richmond, CA, USA).

### Statistical analysis

Data are presented as mean ± standard deviation and were analyzed by the Student’s t test or one-way analysis of variance followed by Tukey post hoc test. The Mann–Whitney *U* test was used to analyze differences of α-synuclein expression in benign, atypical, and anaplastic meningiomas. *P* values  < 0.05 were considered statistically significant.

## Results

### Upregulation of α-synuclein in atypical and anaplastic meningiomas

To check the involvement of α-synuclein in meningioma progression, we examined its expression in 44 meningioma samples. qRT-PCR analysis showed increased abundance of α-synuclein mRNA in atypical (*P* = 0.0067) and anaplastic (*P* = 0.0035) meningiomas (Fig. 1a). We also measure the level of α-synuclein in human malignant meningioma cell lines. The mRNA expression of α-synuclein was significantly increased in IOMM-Lee cells and to a greater extent in CH-157MN cells, when compared to primary meningeal cells (*P* < 0.05; Fig. 1b). Therefore, in this study, IOMM-Lee cells were used in α-synuclein knockdown experiments, while CH-157MN cells were used in α-synuclein overexpression experiments.

**Fig. 1:** Upregulation of α-synuclein in atypical and anaplastic meningiomas. **a** qRT-PCR analysis of α-synuclein mRNA in benign, atypical, and anaplastic meningiomas. **b** Measurement of α-synuclein mRNA in normal meningeal cells and IOMM-Lee and CH-157MN meningioma cells. *P < 0.05 versus normal meningeal cells

### Knockdown of α-synuclein reduces cell proliferation and colony formation and increases apoptosis in IOMM-Lee meningioma cells

To determine the biological significance of α-synuclein dysregulation in meningioma, RNA interfering technology was employed to knock down its expression. As shown in Fig. 2a, delivery of specific α-synuclein shRNA resulted in about 85% decline in α-synuclein mRNA levels in IOMM-Lee cells (*P* < 0.05 vs. control shRNA-transfected cells). Consistently, the α-synuclein protein levels were also decreased in IOMM-Lee cells transfected with α-synuclein shRNA (Fig. 2a). Downregulation of α-synuclein inhibited cell proliferation by 42% in IOMM-Lee cells, as determined by BrdU incorporation assay (Fig. 2b). Colony formation assays further demonstrated that knockdown of α-synuclein led to a 65% reduction in the number of colonies after incubation for 10 days (Fig. 2c). Additionally, the percentage of apoptotic cells was significantly greater in the α-synuclein shRNA group than in the control shRNA group (26.9 ± 2.3% vs. 4. 8 ± 1.2%, *P* < 0.05; Fig. 2d).

The article "Alpha-synuclein contributes to malignant progression of human meningioma via the Akt/mTOR pathway" was published in 2016. Journal: Cancer Cell Int.

**Fig. 2:** Knockdown of α-synuclein (α-Syn) reduces cell proliferation and colony formation and increases apoptosis in meningioma cells. **a** Measurement of α-Syn mRNA and protein levels in IOMM-Lee meningioma cells transfected with control or α-Syn shRNA. **b** BrdU incorporation assay was performed to determine cell proliferation in IOMM-Lee cells transfected with control or α-Syn shRNA. **c** Colony formation assay. IOMM-Lee cells transfected with control or α-Syn shRNA were allowed to form colonies for 10 days. *Top* representative dishes. *Bottom* quantification of colony formation. **d** Apoptosis was quantified by flow cytometry. *Top* representative dot plots of cells stained with Annexin-V and PI. *Bottom* quantitative data from three independent experiments. *P < 0.05 versus cells transfected with control shRNA

### Silencing of α-synuclein attenuates IOMM-Lee cell migration and invasion

Next, we investigated the effect of silencing of α-synuclein on the migration and invasion of IOMM-Lee cells. Wound-healing assay demonstrated that the percentage of wound closure was significantly lower in the α-synuclein-depleted group than in the control group, after incubation for 48 h (*P* < 0.05; Fig. 3a). Transwell invasion assay showed that the number of invaded cells was reduced by 44% after transfection with α-synuclein shRNA, compared with the control group (*P* < 0.05; Fig. 3b). These results indicate that α-synuclein is implicated in the invasiveness of meningioma cells.

**Fig. 3:** Silencing of α-synuclein (α-Syn) attenuates IOMM-Lee cell migration and invasion. **a** In vitro wound-healing assay. IOMM-Lee cells transfected with control or α-Syn shRNA were subjected to in vitro wound-healing assay. *Left* representative images of wounded monolayers at 0 and 48 h after scratching. *Right* quantitative data from three independent experiments. **b** Transwell invasion assay. *Left* representative images of cells that invaded through the Matrigel-coated insert. *Right* quantitative data from three independent experiments. *P < 0.05 versus cells transfected with control shRNA

The article "Alpha-synuclein contributes to malignant progression of human meningioma via the Akt/mTOR pathway" was published in 2016. Journal: Cancer Cell Int.

### The Akt/mTOR pathway is inhibited in α-synuclein-depleted IOMM-Lee cells

At the molecular level, we noted that the phosphorylation levels of mTOR and its substrates p70S6K and 4EBP, as well as Akt were significantly reduced in α-synuclein-depleted IOMM-Lee cells (Fig. 4). However, total amounts of mTOR, p70S6K, 4EBP, and Akt protein were not altered by α-synuclein silencing.

**Fig. 4:** The Akt/mTOR pathway is inhibited in α-synuclein (α-Syn)-depleted cells. Western blot analysis of indicated proteins in IOMM-Lee cells transfected with control or α-Syn shRNA. *Left* representative Western blots from three independent experiments. *Right* quantitative analysis of the phosphorylated/total protein levels. *P < 0.05

### Overexpression of α-synuclein promotes CH-157MN cell growth and invasion

To complement the knockdown experiments, overexpression studies were also conducted. Enforced expression of α-synuclein (Fig. 5a) was found to accelerate cell proliferation (Fig. 5b) and colony formation (Fig. 5c) in CH-157MN meningioma cells. Moreover, α-synuclein-overexpressing CH-157MN cells exhibited a 2.1-fold increase in invasiveness, compared to empty vector-transfected cells (Fig. 5d). These observations underscore the importance of α-synuclein in the aggressiveness of meningioma cells.

**Fig. 5:** Overexpression of α-synuclein (α-Syn) promotes CH-157MN cell growth and invasion. **a** Western blot analysis of α-Syn protein levels in CH-157MN cells transfected with vector (control) or α-Syn-expressing plasmid. *Top* representative Western blots from three independent experiments. *Bottom* quantitative analysis of the α-Syn protein levels. **b** BrdU incorporation assay was performed to determine cell proliferation in CH-157MN cells. **c** Colony formation assay. CH-157MN cells transfected with vector or α-Syn-expressing plasmid were allowed to form colonies for 10 days. *Top* representative dishes. *Bottom* quantification of colony formation. **d** Transwell invasion assay. *Top* representative images of cells that invaded through the Matrigel-coated insert. *Bottom* quantitative data from three independent experiments. *P < 0.05 versus cells transfected with vector

### Depletion of α-synuclein retards tumor growth in a mouse xenograft model

Finally, we studied in vivo therapeutic potential of depletion of α-synuclein in controlling meningioma growth. To this end, IOMM-Lee cells stably transfected with α-synuclein shRNA or control shRNA were subcutaneously injected into nude mice, and tumor growth was assessed. Notably, α-synuclein-depleted IOMM-Lee cells formed significantly smaller xenograft tumors from 10 days after cell injection (Fig. 6a). Final tumor weight was only 38% of the control group (*P* < 0.05; Fig. 6b). Immunohistochemical analysis confirmed that α-synuclein-depleted tumors had a significantly lower percentage of Ki-67-positive cells than control counterparts (*P* < 0.05; Fig. 6c).

The article "Alpha-synuclein contributes to malignant progression of human meningioma via the Akt/mTOR pathway" was published in 2016. Journal: Cancer Cell Int.

**Fig. 6:** Depletion of α-synuclein (α-Syn) retards tumor growth in a mouse xenograft model. IOMM-Lee cells stably transfected with α-Syn shRNA or control shRNA were subcutaneously injected into nude mice (n = 4) and tumor volumes were measured every 5 days. **a** Tumor growth curves based on tumor volumes. **b** Tumors were resected and weighed at 25 days after cell injection. **c** Immunohistochemical staining for Ki-67 in the tumors. *Top* representative images of tissue sections stained for Ki-67. *Bottom* quantitative analysis of Ki-67-positive cells. *Scale bars* 100 μm. *P < 0.05

## Discussion

Members of the synuclein family have been associated with the development of certain tumors [13]. It was reported that γ-synuclein expression is dysregulated in oral squamous cell carcinoma [14], esophageal cancer [15], and breast cancer [16]. The α-synuclein protein shows distinct tissue distributions and is predominantly expressed in brain tumors and melanomas [8, 9, 17]. In agreement with a previous study [9], we found that α-synuclein expression was very low in benign meningiomas. However, an increased expression of α-synuclein was observed in atypical and anaplastic meningiomas, suggesting its implication in the malignant progression of meningiomas.

To explore the biological relevance of α-synuclein upregulation, we performed loss- and gain-of-function studies. The results showed that downregulation of α-synuclein inhibited cell proliferation and colony formation in IOMM-Lee meningioma cells, whereas overexpression of α-synuclein led to opposite outcomes in CH-157MN meningioma cells. Moreover, knockdown of α-synuclein significantly triggered apoptotic death in IOMM-Lee cells, suggesting that α-synuclein is required for the growth and survival of meningioma cells. In vivo studies confirmed that α-synuclein contributes to tumorigenicity of meningioma cells. It has been documented that extracellular α-synuclein at nanomolar concentrations promotes dopaminergic neuronal survival [18]. However, secreted α-synuclein from SH-SY5Y neuroblastoma cells exert detrimental effects on the survival of recipient neuronal cells [19]. Another study demonstrated that overexpression of α-synuclein causes non-apoptotic death in human neuronal cells [20]. These studies, combined with our findings, suggest that α-synuclein has distinct roles in the regulation of cell survival in different biological settings.

The article "Alpha-synuclein contributes to malignant progression of human meningioma via the Akt/mTOR pathway" was published in 2016. Journal: Cancer Cell Int.

In addition to regulation of cell proliferation and survival, our data showed that α-synuclein also modulates the migration and invasion of meningioma cells. We observed that α-synuclein silencing suppressed the motility and invasiveness of IOMM-Lee meningioma cells. In contrast, overexpression of α-synuclein facilitated the invasion of CH-157MN meningioma cells. The pro-invasive capacity of α-synuclein provides a biological explanation for its upregulation in atypical and anaplastic meningiomas. Although there is few evidence for α-synuclein-mediated cell invasiveness, γ-synuclein has been shown to promote cell migration and invasion in different types of tumor cells such as oral squamous cell carcinoma [12], breast cancer [21], and gastric cancer [22].

Activation of the Akt/mTOR pathway is involved in the development and progression of meningioma [3, 4]. Fibroblast growth factor receptor-3 was found to induce the proliferation of meningioma cells via activation of the phosphoinositide 3 kinase-Akt-PRAS40-mTOR and STAT3 pathways [23]. Pharmacological inhibition of mTOR signaling was reported to impair meningioma growth in mouse models [24]. Inhibition of Akt activation accounts for growth reduction and apoptosis induction by depletion of astrocyte elevated gene-1 in human meningioma cells [25]. Notably, our data showed that α-synuclein silencing significantly decreased the phosphorylation of Akt, mTOR, p70S6K, and 4EBP in IOMM-Lee cells, which provides a mechanistic explanation for the regulation of aggressive phenotypes of meningioma cells by α-synuclein.

## Conclusions

In conclusion, α-synuclein is upregulated in atypical and anaplastic meningiomas compared to benign tumors and α-synuclein upregulation contributes to the aggressive behavior of meningioma cells via the Akt/mTOR pathway. Thus, α-synuclein represent a potential therapeutic target against malignant meningiomas.

## Abbreviations

BrdU: 5-bromo-2′-deoxyuridine
DMEM: Dulbecco’s modified Eagle medium
FBS: fetal bovine serum
PD: Parkinson’s disease
qRT-PCR: quantitative real-time PCR
shRNA: small hairpin RNA

## References

[1] Backer-Grøndahl T, Moen BH, Torp SH (2012). The histopathological spectrum of human meningiomas. Int J Clin Exp Pathol.

[2] Pećina-Šlaus N, Kafka A, Lechpammer M (2016). Molecular genetics of intracranial meningiomas with emphasis on canonical Wnt signalling. Cancers.

The article "Alpha-synuclein contributes to malignant progression of human meningioma via the Akt/mTOR pathway" was published in 2016. Journal: Cancer Cell Int.

[3] El-Habr EA, Levidou G, Trigka EA, Sakalidou J, Piperi C, Chatziandreou I (2014). Complex interactions between the components of the PI3K/AKT/mTOR pathway, and with components of MAPK, JAK/STAT and Notch-1 pathways, indicate their involvement in meningioma development. Virchows Arch.

[4] Johnson MD, O’Connell M, Vito F, Bakos RS (2009). Increased STAT-3 and synchronous activation of Raf-1-MEK-1-MAPK, and phosphatidylinositol 3-Kinase-Akt-mTOR pathways in atypical and anaplastic meningiomas. J Neurooncol.

[5] Armando V, Antonio G, Giovanni F, Maurizio I, Ida RM, Andrea G (2016). Parkinson’s disease: autoimmunity and neuroinflammation. Autoimmun Rev.

[6] Matsuo Y, Kamitani T (2010). Parkinson’s disease-related protein, α-synuclein, in malignant melanoma. PLoS ONE.

[7] Surguchov A (2016). Parkinson’s disease: assay of phosphorylated α-synuclein in skin biopsy for early diagnosis and association with melanoma. Brain Sci.

[8] Pan T, Zhu J, Hwu WJ, Jankovic J (2012). The role of α-synuclein in melanin synthesis in melanoma and dopaminergic neuronal cells. PLoS ONE.

[9] Kawashima M, Suzuki SO, Doh-ura K, Iwaki T (2000). α-Synuclein is expressed in a variety of brain tumors showing neuronal differentiation. Acta Neuropathol.

[10] Louis DN, Ohgaki H, Wiestler OD, Cavenee WK, Burger PC, Jouvet A (2007). The 2007 WHO classification of tumours of the central nervous system. Acta Neuropathol.

[11] Alvarez-Erviti L, Seow Y, Schapira AH, Rodriguez-Oroz MC, Obeso JA, Cooper JM (2013). Influence of microRNA deregulation on chaperone-mediated autophagy and α-synuclein pathology in Parkinson’s disease. Cell Death Dis.

[12] He X, Zhou C, Zheng L, Xiong Z (2014). Overexpression of MTA1 promotes invasiveness and metastasis of ovarian cancer cells. Ir J Med Sci.

[13] Surguchov A (2015). Intracellular dynamics of synucleins: “here, there and everywhere”. Int Rev Cell Mol Biol.

[14] Cheng JC, Chiang MT, Lee CH, Liu SY, Chiu KC, Chou YT (2016). γ-Synuclein expression is a malignant index in oral squamous cell carcinoma. J Dent Res.

[15] Tastekin D, Kargin S, Karabulut M, Yaldız N, Tambas M, Gurdal N (2014). Synuclein-γ predicts poor clinical outcome in esophageal cancer patients. Tumour Biol.

[16] Wu K, Huang S, Zhu M, Lu Y, Chen J, Wang Y (2013). Expression of synuclein γ indicates poor prognosis of triple-negative breast cancer. Med Oncol.

[17] Fung KM, Rorke LB, Giasson B, Lee VM, Trojanowski JQ (2003). Expression of α-, β-, and γ-synuclein in glial tumors and medulloblastomas. Acta Neuropathol.

[18] Kim JY, Jeon BS, Kim HJ, Ahn TB (2013). Nanomolar concentration of α-synuclein enhances dopaminergic neuronal survival via Akt pathway. Neural Regen Res.

The article "Alpha-synuclein contributes to malignant progression of human meningioma via the Akt/mTOR pathway" was published in 2016. Journal: Cancer Cell Int.

[19] Emmanouilidou E, Melachroinou K, Roumeliotis T, Garbis SD, Ntzouni M, Margaritis LH (2010). Cell-produced α-synuclein is secreted in a calcium-dependent manner by exosomes and impacts neuronal survival. J Neurosci.

[20] Vekrellis K, Xilouri M, Emmanouilidou E, Stefanis L (2009). Inducible over-expression of wild type α-synuclein in human neuronal cells leads to caspase-dependent non-apoptotic death. J Neurochem.

[21] Zhuang Q, Liu C, Qu L, Shou C (2015). Synuclein-γ promotes migration of MCF7 breast cancer cells by activating extracellular-signal regulated kinase pathway and breaking cell–cell junctions. Mol Med Rep.

[22] Wang Y, Liu X, Zhang H, Sun L, Zhou Y, Jin H (2014). Hypoxia-inducible lncRNA-AK058003 promotes gastric cancer metastasis by targeting γ-synuclein. Neoplasia.

[23] Johnson MD, O’Connell MJ, Pilcher W, Reeder JE (2010). Fibroblast growth factor receptor-3 expression in meningiomas with stimulation of proliferation by the phosphoinositide 3 kinase-Akt pathway. J Neurosurg.

[24] Pachow D, Andrae N, Kliese N, Angenstein F, Stork O, Wilisch-Neumann A (2013). mTORC1 inhibitors suppress meningioma growth in mouse models. Clin Cancer Res.

[25] Park KJ, Yu MO, Song NH, Kong DS, Park DH, Chae YS (2015). Expression of astrocyte elevated gene-1 (AEG-1) in human meningiomas and its roles in cell proliferation and survival. J Neurooncol.

